# Qingchang Wenzhong Decoction Alleviates DSS-Induced Inflammatory Bowel Disease by Inhibiting M1 Macrophage Polarization *In Vitro* and *In Vivo*

This article has been retracted.

**DOI:** 10.1155/2022/9427076

**Published:** 2022-08-25

**Authors:** Qiongqiong Lu, Junxiang Li, Panghua Ding, Tangyou Mao, Lei Shi, Zhongmei Sun, Xiang Tan, Hui Jiang, Junying Dong, Yalan Li, Xiaojun Yang, Rui Shi

**Affiliations:** ^1^Graduate School, Beijing University of Chinese Medicine, Beijing, China; ^2^Department of Gastroenterology, Chongqing Traditional Chinese Medicine Hospital, Chongqing, China; ^3^Department of Gastroenterology, Dongfang Hospital, Beijing University of Chinese Medicine, Beijing, China

## Abstract

**Background:**

An imbalance of macrophage M1/M2 polarization significantly influences the pathogenesis of inflammatory bowel disease. Qingchang Wenzhong decoction (QCWZD) has a proven therapeutic effect on patients with inflammatory bowel disease (IBD) and can significantly inhibit the inflammatory response in mice with colitis. However, its effect on macrophages during IBD treatment remains nebulous. *Aim of the Study*. Explore the mechanism underlying QCWZD effects in a dextran sulfate sodium (DSS)-induced colitis mouse model in vivo and RAW264.7 cell in vitro by observing macrophage polarization dynamics.

**Methods:**

The main active components of QCWZD were determined using high-performance liquid chromatography. Surface marker expression on M1-type macrophages was analyzed using flow cytometry and immunofluorescence. The effect on inducible nitric oxide synthase (iNOS), interleukin-6 (IL-6), and tumor necrosis factor-*α* (TNF-*α*) released by M1 type macrophages was determined using ELSA and RT-PCR. The expression of key proteins in the JAK2/STAT3 signaling pathway was analyzed using western blotting. QCWZD cytotoxicity in macrophages was measured using CCK8 and Annexin V-FITC/PI assays.

**Results:**

The main active components of QCWZD were berberine chloride, coptisine chloride, epiberberine chloride, gallic acid, ginsenoside Rg1, ginsenoside Rb1, indigo, indirubin, notoginsenoside R1, palmatine chloride, and 6-curcumin. QCWZD markedly alleviated DSS-induced colitis in mice, as revealed by the rescued weight loss and disease activity index, attenuated the colonic shortening and mucosal injury associated with the inhibition of M1 macrophage polarization and expression of related cytokines, such as IL-6 and TNF-*α*, *in vivo* and *in vitro*. Furthermore, QCWZD decreased the iNOS, JAK2, and STAT3 levels *in vivo* and *in vitro*, regulating the JAK2/STAT3 signaling pathway.

**Conclusion:**

QCWZD administration improves intestinal inflammation by inhibiting M1 macrophage polarization. The JAK2/STAT3 signaling pathway may mediate the effects of QCWZD on M1 macrophage polarization in colitis treatment. This study presents a novel macrophage-mediated therapeutic strategy for the treatment of IBD.

## 1. Introduction

Inflammatory bowel disease (IBD), of unknown etiology, is a chronic inflammatory gastrointestinal disorder. Crohn's disease (CD) and ulcerative colitis (UC) are two types of IBD. Primary symptoms of UC include hemorrhagic diarrhea, weight loss, and abdominal cramps [1–3] with lesions restricted to the colon and rectum. The reported incidence of IBD has risen significantly in recent decades [4]. To date, the available therapeutic strategies for IBD mainly comprise the administration of salicylates, steroids, immunomodulators, and biological agents [5]. However, IBD symptom recurrence in remission and adverse drug reactions, such as autoimmunity, liver toxicity, malignancies, and opportunistic infections, caused by long-term maintenance therapy remain major challenges [6]. Furthermore, IBD might require colectomy as a treatment option [7, 8]. Therefore, it is necessary to develop novel and safe therapeutic strategies for IBD.

Macrophages play a significant role in the innate immune response, which identifies and removes bacteria and foreign bodies. They are also key regulators of intestinal microenvironment homeostasis, perform inflammation-promoting functions in injured colon tissue via phenotypic polarization, and are intimately involved in IBD pathogenesis [9, 10]. Stimulated by different factors or substrates, macrophages can be activated and polarized into the inflammation-promoting M1 subtype [11, 12]. M1 macrophage polarization is initiated by immune responses to characteristic components of bacteria or interferon-*γ* (IFN-*γ*) [13]. M1 macrophages exhibit high expression of proinflammatory factors, mainly interleukin-6 (IL-6) and tumor necrosis factor-*α* (TNF-*α*) [14]. Murine M1 macrophages can co-express F4/80 and CD16/32 [15, 16]. In dextran sulfate sodium- (DSS-) induced colitis, M1 macrophages are involved in disease progression by producing proinflammatory cytokines, leading to mucosal barrier lesions [17]. Therefore, the targeted manipulation of M1-type macrophage polarization may be an effective strategy for the treatment of UC.

Traditional Chinese medicines, particularly herbal medicines, have recently been used in patients with IBD [18, 19]. Qingchang Wenzhong Decoction (QCWZD) is a traditional Chinese empirical herbal prescription used in the Department of Gastroenterology, Dongfang Hospital Beijing University of Chinese Medicine (BUCM; Beijing, China) for many years. It has been proved to relieve the clinical symptoms in patients with UC [20, 21], reduce inflammatory responses, improve intestinal barrier functions, and regulate the microorganism population in DDS-induced UC rat models [22–24]. However, the effects of QCWZD on macrophages in the treatment of IBD remain unclear. In this study, we investigated the mechanism underlying the effect of QCWZD on a DSS-induced colitis mouse model *in vivo* and RAW264.7 cell *in vitro* by observing the dynamic changes of macrophage polarization.

## 2. Materials and Methods

### 2.1. Drugs and High-Performance Liquid Chromatography (HPLC) Analysis

QCWZD, composed of the following eight herbs: 6 g Huang Lian (*Coptis chinensis* Franch.), 10 g Pao Jiang (*Zingiber officinale* Roscoe), 9 g Ku Shen (*Sophora flavescens* Aiton), 3 g Qing Dai (*Strobilanthes cusia* (Nees) Kuntze), 15 g Di Yu Tan (*Sanguisorba officinalis* L.), 6 g Mu Xiang (*Aucklandia costus* Falc.), 6 g San Qi (*Panax notoginseng* (Burkill) F.H. Chen), and 6 g Gan Cao (*Glycyrrhiza glabra* L.), was supplied by Dongfang Hospital, Beijing University of Chinese Medicine (BUCM), Beijing, China. The herbs were extracted, using decoction, condensation, and dehydration, and made into granules. Herb processing was conducted by Beijing Kangrentang Pharmaceutical (Beijing, China). All processes were performed based on the guide to Good Manufacturing Practice for Drugs to ensure optimal drug quality. HPLC (Waters 2695-2998 series HPLC system) analyses were conducted to identify the primary chemical components of QCWZD [20].

The following chemicals were used as measurement standards: berberine chloride, coptisine chloride, epiberberine chloride, gallic acid, ginsenoside Rb1, ginsenoside Rg1, indigo, indirubin, notoginsenoside R1, palmatine chloride, and 6-curcumin. All chemicals were supplied by the National Medical Products Administration (Beijing, China). Chromatographic separation was carried out using Reprosil-Pur Basic-C18 (5 *μ*m, 4.6 × 250 mm, 100 A°) with a mobile phase of acetonitrile (solvent A) and aqueous solution of 0.1% formic acid (FA) (solvent B). The injection volume was set at 10 *μ*L while the detector wavelength was set at 280 nm for 6-curcumin, 270 nm for gallic acid, 345 nm for berberine chloride, coptisine chloride, epiberberine chloride, and palmatine chloride, 292 nm for indigo and indirubin, and 203 nm for ginsenoside Rb1, ginsenoside Rg1, and notoginsenoside R1.

### 2.2. Animals

Animal experiments were accredited by the Animal Ethics Committee of BUCM and were performed following the guidelines of the Regulations of Beijing Laboratory Animal Management. Twenty female C57BL/6 mice (18–20 g; 6–8 weeks old) were supplied by Beijing Vital River Laboratory Animal Technology (SCXK-2016-0006; Beijing, China). Mice were housed in specific pathogen-free (SPF) facilities and exposed to ambient photoperiod, temperatures of 20–24°C, and humidity levels of 50%–60%, with free access to standard chow and sterile water.

### 2.3. Cells

RAW264.7 cells were purchased from the National Biomedical Experimental Cell Resource Bank (1101MOU-PUMC000146, Beijing, China).

### 2.4. Grouping and Administration

Mice were maintained at the SPF animal facilities of BUCM. An acute colitis mouse model was established by administration of 2.5% (w/v) DSS (MP Biomedicals, Santa Ana, CA, USA) supplied through drinking water for seven days. During the modeling period, the stool quality and occult blood or blood in the stool were monitored to determine if the modeling was successful. Mice were divided into control, DSS (DSS), DSS + QCWZD (DQ), and DSS + mesalazine (DM) groups (*n* =6/group). Control mice received sterile water, whereas those in the DSS, DQ, and DM groups received sterile water containing 2.5% DSS for seven days. During this 7-day treatment period, the control and DSS-treated mice received treatment in 0.2 mL sterile tap water. Mice in the DQ group received 0.2 mL of 9.25 g/kg QCWZD (the animal equivalent dose was determined by calculating the ratio of the experimental animal body surface area to the human body surface area), while mice in the DM group received 0.2 mL of 0.61 g/kg mesalazine (Ethypharm, Shanghai, China). Sterile tap water was provided for two additional days before sacrifice. All mice were sacrificed after inhalation anesthesia with isoflurane (half lethal dose [LD_50_] =5080 *μ*L/kg) on day 9 and samples were collected for further analysis.

### 2.5. Disease Activity Index (DAI) Analysis

The DAI was evaluated daily based on previously defined criteria including body weight loss, stool consistency, and rectal bleeding [25].

### 2.6. Evaluation of Colonic Damage

Colonic samples were kept in formalin solution (10%), embedded in paraffin, sliced (5 *μ*m), and stained with hematoxylin and eosin (H&E). Lesion scores based on the histochemical analysis were determined based on previously used criteria [26]. Both immune cell infiltration and tissue lesions were considered for determining the histological scores. The following scoring system was used for immune cell infiltration evaluation: 0, no infiltration; 1, positive immune infiltration in the lamina propria (LP); 2, positive immune infiltration in submucosa; and 3, transmural immune infiltration. The following scoring system was used for tissue lesion evaluation: 0, no mucosal damage; 1, mild epithelial damage; 2, moderate erosions or focal ulceration; 3, severe mucosal lesion with heavy ulceration extending to the bowel wall.

### 2.7. Cell Culture and M1 Macrophage Induction

RAW264.7 cells were cultured in Dulbecco's Modified Eagle Medium (DMEM) (ThermoFisher Scientific, Waltham, MA, USA) supplemented with 10% fetal bovine serum (ThermoFisher Scientific), 100 U/mL penicillin (ThermoFisher Scientific), and 100 *μ*g/mL streptomycin (ThermoFisher Scientific). M1 polarization of RAW264.7 cells was induced by incubating cells with 100 ng/mL lipopolysaccharide (LPS) and 10 ng/mL IFN-*γ* (from *Escherichia coli*, Sigma, St. Louis, MO, USA) for 24 h. QCWZD treatment was conducted 2 h before the stimulation with LPS and IFN-*γ*.

### 2.8. Immunofluorescence

Colon tissue paraffin sections (5 *μ*m) were dewaxed and rehydrated. Antigen retrieval was performed in an ethylenediaminetetraacetic acid solution. Tissue sections were blocked in bovine serum albumin for 30 min and incubated with the following primary antibodies: anti-F4/80 (1 : 1,200, Servicebio, Wuhan, China) and anti-CD16/32 (1 : 200, TONBO biosciences, San Diego, CA, USA). Phosphate buffer saline was used to wash (x3) the tissue sections. Secondary Alexa Fluor 488 or CY3 conjugated antibodies (Servicebio, Wuhan, China) were then incubated with the tissue sections for 1 h [15]. The cell nuclei were stained with 4′,6-diamidino-2-phenylindole for 10 min. Confocal laser scanning microscopy was used for image capture.

### 2.9. RNA Extraction and Real-Time Reverse Transcription-Quantitative Polymerase Chain Reaction (RT-qPCR)

Total RNA was extracted from colon tissue and RAW264.7 cells using TRIzol (Invitrogen, Waltham, MA, USA), reverse transcribed to cDNA, added primers (Sangon Biotech, Shanghai, China) (the sequence is shown in Table 1), and used for RT-qPCR, performed on the ABI PRISM 7500 detection system (Applied Biosystems, Waltham, MA, USA) using the Fast SYBR® Green Master Mix (ThermoFisher Scientific). The amplification program included a denaturation step at 95°C for 2 min, and 35 cycles of 10 s at 95°C, 30 s at 62°C, followed by 30 s at 72°C. The relative mRNA expression levels were calculated using the 2^-*ΔΔ*CT^ method.

### 2.10. Enzyme-Linked Immunosorbent Assay (ELISA)

Following blood sample collection, the levels of IL-6 (Biolegend, 431307) and TNF-*α* (Biolegend, 430907) were measured using ELISA kits following the manufacturer's instructions.

### 2.11. Western Blotting

Samples were collected and lysed in a precooled RIPA protein extraction reagent (TDY, WB0003, Beijing, China) containing a protease inhibitor. The lysate was electrophoresed, and the proteins were electro-transferred from the gel onto a nitrocellulose membrane (Millipore Corp., HATF00010, NJ, USA) at room temperature (20°C). The membrane was blocked with 5% skimmed milk and subsequently incubated overnight with the primary antibody at 4°C. The following primary antibodies were used: anti-JAK2 antibody (Abcam, ab108596, Cambridge, UK, 1 : 1,000, 130 kDa), anti-JAK2 (phospho Y1007 + Y1008) antibody (Abcam, ab32101, 1 : 2,000, 130 kDa), and anti-STAT3 antibody (Abcam, ab68153, 1 : 1,000, 88 kDa), and anti-STAT3 (phospho Y705) antibody (Abcam, ab267373, 1 : 1,000, 88 kDa). The membrane was then incubated with a suitable horseradish peroxidase-conjugated secondary antibody and subsequently with the substrate. The protein bands were visualized, and densitometry was conducted using the Total Lab Quant V 11.5 software (Newcastle upon Tyne, UK).

### 2.12. Cytotoxicity Test

When RAW264.7 cells reached 90% confluence, they were digested with 0.25% trypsin, diluted with complete medium, and counted. Then, they were inoculated in 96-well plates at a density of 8 × 10^4^ cells/100 *μ*L/well and cultured in a constant temperature incubator with 5% CO_2_ at 37°C for 24 h. The culture medium was then discarded and 100 *μ*L filtered QCWZD solution was added to each well at different concentrations (1, 0.5, 0.25, 0.125, 0.0625, or 0.03125 mg/mL). Control cells were treated with 100 *μ*L basal medium. After 24 h of culture, the medium was discarded and 90 *μ*L basal medium and 10 *μ*L CCK8 solution (Solarbio, JP) were added to each well, and cells were cultured in an incubator for another 1-4 h. Next, the OD value of each well was measured at 450 nm using a full-wavelength scanning microplate reader, and the survival rate was calculated.

### 2.13. Annexin V-FITC/PI Detection

When RAW264.7 cells reached 90% confluence, they were digested with 0.25% trypsin, resuspended in complete medium and divided into bottles. Then, the cells were treated with different concentrations of filtered QCWZD solution (0, 0.25, 0.125, or 0.0625 mg/mL) and grown at 37°C. Control cells were treated with complete medium. The culture medium was discarded and cells were digested with EDTA-free trypsin. Digestion was terminated with complete medium. The cells were collected using centrifugation at 4°C for 10-15 min at 1000 rpm, resuspended in precooled 1 × PBS (4°C), and centrifuged for 10-15 min at 1000 rpm, followed by washing. A total of 300 *μ*L 1 × Binding Buffer was added and the cells were resuspended by air blowing. Then, 5 *μ*L Annexin V-FITC was added, followed by incubation at room temperature for 15 min. A total of 5 *μ*L PI was added before staining, and 200 *μ*L 1 × Binding Buffer was added for testing.

### 2.14. Flow Cytometry

Collect RAW264.7 cells, F4/80, and CD16/32 antibodies were added and incubated at 4°C in the dark for 30 min to stain the cell membrane surface. Next, the cells were washed, centrifuged, and resuspended, and a flow cytometer (BD, BC, NJ, USA) was used for detection. Data analysis was performed using Flowjo VX10. The following fluorochrome-labelled antibodies were used for the staining of macrophages: CD16/32 allophycocyanin (Biolegend, San Diego, CA, USA; 101323) and F4/80 fluorescein isothiocyanate (Biolegend; 123107). The cell type identification criteria were as follows: F4/80^+^ defined macrophages and F4/80^+^CD16/32^+^ the M1 subtype.

### 2.15. Statistical Analysis

The SPSS 22.0 software (IBM Corp., Chicago, NY, USA) was used for the statistical analysis. Data are presented as the mean ± SD for independent experiments. Two group comparisons were assessed by one-way analysis of variance (ANOVA) followed by the least significant difference (LSD) post hoc test. A *P* value of <0.05 was considered statistically significant.

## 3. Results

### 3.1. Qualitative and Quantitative HPLC Analysis of QCWZD

Quantitative HPLC analysis was conducted for QCWZD. The main active components of QCWZD against experimental colitis were berberine chloride, coptisine chloride, epiberberine chloride, gallic acid, ginsenoside Rb1, ginsenoside Rg1, indigo, indirubin, notoginseno side R1, palmatine chloride, and 6-curcumin. Satisfying degrees of separation and methodological investigations were observed (Figures 1(a)–1(e)). The amounts of major indices in QCWZD were calculated according to standards (Table 2).

### 3.2. QCWZD Treatment Ameliorates DSS-Induced Colitis

Treatment procedures are demonstrated in Figure 2(a). As shown in Figures 2(b)–2(e), the DSS treatments caused colonic inflammatory reactions, as revealed by the body weight loss, increased DAI scores, and colonic shortening. As expected, supplementation with QCWZD and mesalazine partly attenuated the above-mentioned DSS treatment-induced alterations. Histological analyses of the colon tissue from DSS-treated mice demonstrated severe mucosal necrosis and inflammation infiltration. However, the pathological damage (Figures 2(f) and 2(g)) was to a certain degree attenuated by QCWZD treatment. Collectively, our results suggest that QCWZD treatment significantly ameliorates DSS-induced intestinal inflammation and colonic damage.

### 3.3. Effects of QCWZD on M1-Type Macrophages and Associated Inflammatory Cytokines

To explore the effects of QCWZD on M1 macrophage polarization, immunofluorescence was performed. As observed in Figure 3(a), the intestinal inflammation induced by DSS treatment increased the number of inflammatory M1 macrophages (identified by F4/80^+^CD16/32^+^) in mice. The inducible nitric oxide synthase (iNOS) is an important marker of M1 macrophage activation [27] RT q-PCR demonstrated significant upregulation of iNOS by DSS treatment (*P* < 0.05; Figure 3(b)). However, QCWZD reversed this effect and significantly decreased the frequency of F4/80^+^CD16/32^+^ cells (*P* < 0.05) (Figures 3(a) and 3(b)). Another manifestation of DSS-induced colitis was the increased levels of proinflammatory factors, including IL-6 and TNF-*α*, primarily secreted by M1 macrophages [28]. As expected, a significant increase in the serum levels of IL-6 and TNF-*α* was found in DSS-treated mice (both *P* < 0.01), whereas mice treated with QCWZD showed a significant attenuation of these manifestations (*P* < 0.05 and *P* < 0.01, respectively; Figures 3(c) and 3(d)). RT-qPCR analysis of the IL-6 and TNF-*α* levels yielded similar results (*P* < 0.05 and *P* < 0.01, respectively; Figures 3(e) and 3(f)). The above results collectively demonstrate the inhibitory effects of QCWZD in regulating macrophage polarization to M1-like subtype and reducing inflammatory responses in DSS-induced colitis.

### 3.4. QCWZD Regulates JAK2/STAT3 Signaling Pathway

To determine if QCWZD regulates the JAK2/STAT3 signaling pathway, we assessed the expression of key proteins in the JAK2/STAT3 signaling pathway. We found that QCWZD reduced the ratios of p-JAK2/JAK2 and p-STAT3/STAT3 (*P* < 0.01 and *P* < 0.05, respectively; Figures 4(a)–4(d)), thereby exerting a regulatory effect on JAK2/STAT3 signaling. These results indicate that QCWZD may target the JAK2/STAT3 signaling pathway to drive macrophage polarization in colitis treatment.

### 3.5. QCWZD Cytotoxicity in Macrophages

At various concentrations (0.25, 0.125, 0.0625, and 0.03125 mg/mL) of QCWZD, no cytotoxicity was observed in RAW 264.7 cells (Figure 5(a)). Likewise, no significant changes in the apoptosis level of RAW 264.7 cells were observed following QCWZD treatments (0.25, 0.125, and 0.0625 mg/mL) (Figures 5(b) and 5(c)).

### 3.6. QCWZD Treatment Decreases the Number of M1-Like Inflammatory Macrophages in RAW264.7 Cells

The significant roles of QCWZD in the regulation of macrophage polarization associated with the intestinal damages in DSS-treated mice demonstrated *in vivo* were further confirmed by investigating the inhibitory effects of QCWZD on M1 macrophage polarization *in vitro*. RAW264.7 cells were treated with LPS and IFN-*γ* to induce M1 polarization. As revealed using flow cytometry, QCWZD treatments at different concentrations significantly reduced RAW264.7 cell M1 polarization (*P* < 0.01; Figures 6(a) and 6(b)). Furthermore, iNOS expression was significantly rescued in QCWZD-treated RAW264.7 cells (*P* < 0.01; Figure 6(c)). Moreover, ELISA analysis showed that the levels of IL-6 and TNF-*α* were significantly increased in RAW264.7 cells treated with LPS and IFN-*γ* (both *P* < 0.01; Figures 6(d) and 6(e)). However, QCWZD treatment reduced the increased levels of IL-6 and TNF-*α* induced by LPS and IFN-*γ* (*P* < 0.05 and *P* < 0.01, respectively; Figures 6(d) and 6(e)). The above results demonstrate that QCWZD inhibited M1 macrophage polarization and the expression of proinflammatory cytokines, which may explain its inhibitory effect on colitis.

### 3.7. QCWZD Regulates JAK2/STAT3 Signaling Pathway in RAW264.7 Cells

As demonstrated by the aforementioned findings, QCWZD can inhibit JAK2 and STAT3 *in vivo* (Figures 4(a)–4(f)), indicating that the protective effects of QCWZD are potentially associated with the JAK2/STAT3 signaling pathway. To verify if QCWZD can also regulate the JAK2/STAT3 signaling pathway in RAW264.7 cells, the JAK2/STAT3 signaling pathway was investigated *in vitro*. We found that QCWZD treatment significantly inhibited the ratios of phosphorylated JAK2/JAK2 and phosphorylated STAT3/STAT3 (*P* < 0.01 and *P* < 0.05, respectively; Figures 7(c) and 7(d)). Collectively, the above results suggest that QCWZD inhibited the activation of the JAK2/STAT3 signaling pathway.

## 4. Discussion

QCWZD is composed of the following eight herbs: Huang Lian (*Coptis chinensis* Franch.), Pao Jiang (*Zingiber officinale* Roscoe), Ku Shen (*Sophora flavescens* Aiton), Qing Dai (*Strobilanthes cusia* (Nees) Kuntze), Di Yu Tan (*Sanguisorba officinalis* L.), Mu Xiang (*Aucklandia costus* Falc.), San Qi (*Panax notoginseng* (Burkill) F.H. Chen), and Gan Cao (*Glycyrrhiza glabra* L.). The main active components of QCWZD identified using HPLC were berberine chloride, coptisine chloride, epiberberine chloride, gallic acid, ginsenoside Rb1, ginsenoside Rg1, indigo, indirubin, notoginsenoside R1, palmatine chloride, and 6-curcumin, all of which may play major roles in the treatment of UC. Berberine exerts its effect by regulating enteric neurogenic inflammation [29], while gallic acid has been reported to play an anti-inflammatory role in IBD animal models [30]. Indigo naturalis alleviates experimental colitis via altering the gut microbiota [26], while ginsenoside Rd can relieve indomethacin-induced IBD by regulating endogenous intestinal stem cells [31]. These results suggest that QCWZD may alleviate experimental colitis through these active components.

UC is a chronic inflammatory disorder of the gastrointestinal system that seriously impacts human health. The pathogenesis of UC is closely associated with M1 macrophage polarization [15, 32]. During UC pathogenesis, an infiltration of intestinal mucosal inflammatory cells, such as M1 macrophages, is observed with an increase in the level of inflammatory factors secreted by M1 macrophages, along with colonic mucosa hyperemia, edema, and crypt structure disorder [33]. The JAK2/STAT3 pathway is closely related to the regulation of intestinal mucosa tissue inflammation [34] and can regulate the polarization of M1 macrophages [35]. Currently, the methods used for predicting, preventing, and treating this disease remain limited [36, 37]. Therefore, there is an urgent need to develop novel and safe UC treatments. The oral administration of QCWZD is a safe and effective complementary and alternative therapy that can ameliorate the intestinal inflammatory reaction and related colonic lesion in mice. It has low or no toxicity, few side effects, and exhibits definite curative effects [20, 22, 23]. However, the effect of QCWZD on macrophages and the role of the JAK2/STAT3 pathway in IBD treatment remain unclear. In this study, we confirm that QCWZD potently alleviates the intestinal inflammatory reactions and mucosal lesions in mice with DSS-induced colitis, inhibits macrophage polarization toward an M1-like phenotype, and regulates the levels of proteins involved in the JAK2/STAT3 signaling pathway. We propose that QCWZD may inhibit M1 macrophage polarization by regulating the JAK2/STAT3 signaling pathway, thereby mitigating DSS-induced colitis.

The immunofluorescence results showed that QCWZD inhibits macrophage polarization toward the M1-like subtype and contributes to intestinal inflammation remission. Macrophages, which are white blood cells distributed in the colon, are closely associated with IBD development. In response to different local stimuli or various pathophysiological conditions, macrophages may either convert into the inflammation-promoting M1 subtype or the inflammation-inhibiting M2 subtype. During inflammation, macrophages primarily exist in M1-type clusters [38, 39]. M2 macrophages play a protective role in sustaining the homeostasis of intestinal functions and immune responses. At the same time, M1 macrophages can be transformed into M2 macrophages and vice versa in response to specific pathways and molecular actions. With the progress of inflammation, the mechanism regulating the immunoinflammatory response induces the transformation of M1 macrophages to M2 macrophages, which can repair the inflammatory damage and inhibit further inflammation progression [38, 39]. Importantly, M2-type macrophages are cancer-related, and M2-type macrophage studies will be the focus of our subsequent research. Previous studies have revealed that the upregulation of M1 macrophages promotes colitis development [33]. Furthermore, the inhibition of M1 polarization has also been found to alleviate the symptoms of colitis. Moreover, it has been reported that berberine treatments can inhibit the inflammatory responses by regulating macrophage polarization [15]. Lissner et al. found that M1 macrophage infiltration in the intestinal area directly caused epithelial tissue lesions via tight junction disruption and apoptosis induction [40], thereby causing the inflammatory responses associated with IBD. Another study further showed that hemin injection can alleviate intestinal inflammation and repair the damage of intestinal mucosal barriers by correcting abnormal intestinal macrophage polarization both *in vitro* and *in vivo* [33]. Zhou et al. found that Yes-associated protein in macrophages promotes LPS/IFN-*γ*-triggered M1 macrophage activation to aggravate IBD [34]. Therefore, M1 macrophages can drive intestinal inflammation in IBD, and inhibiting M1 macrophage polarization provides a new treatment strategy for IBD. In this study, we demonstrated that QCWZD reduces the levels of proinflammatory factors, such as IL-6 and TNF-*α*, secreted by M1 macrophages both *in vivo* and *in vitro*, thereby alleviating DSS-induced colitis in mice, demonstrating the protective effect of QCWZD in the treatment of IBD. Flow cytometry was used to detect the effect of this traditional Chinese medicine on macrophage apoptosis and observe its cytotoxicity. Our findings showed that QCWZD is not toxic to RAW264.7 cells at a concentration below 0.25 mg/mL.

Our results suggest that QCWZD inhibits M1 macrophage polarization, thereby alleviating the symptoms of DSS-induced colitis. One of the potential underlying mechanisms may involve the JAK2/STAT3 signaling pathway. Studies have confirmed that this pathway is tightly associated with colitis inflammation [41, 42]. For example, *Veronica polita* was found to relieve experimental colitis mediated by inflammatory mediators via suppressing the JAK2/STAT3 signaling pathway [43]. Furthermore, Kong et al. found that hesperetin derivative 12 reduces the levels of M1 macrophages by regulating the JAK2/STAT3 signaling pathway [35]. JAK and STAT are components of an intracellular signaling pathway influencing various cytokines and growth factors [44] associated with immune reactions, cell proliferation, and differentiation, and the regulation of macrophage polarization and activity [39, 45]. The JAK/STAT pathway involves various ligands and their associated receptors, such as JAK and STAT family proteins [46]. Upon binding to cytokines and receptors, a tyrosine phosphorylation cascade is activated, which subsequently leads to JAK activation. For example, following cytokine IL-6 binding to the JAK2 receptor, the inactive JAK2 undergoes a conformational change and is converted into an active tyrosine kinase (p-JAK2), an important step in cytokine-mediated signal transduction [47]. Furthermore, STAT3 signaling plays a pivotal role in the development of many autoimmune diseases [48]. Phosphorylated tyrosine residue (Y705) (p-JAK2) activates and dimerizes STAT3 and the dimerized STAT3 is translocated to the nucleus, where it promotes the transcriptional activation of M1-type macrophage-related genes [49]. The specific underlying mechanism, however, requires further investigation. To verify the effect of QCWZD on the JAK2/STAT3 signaling pathway, we determined the levels of key pathway proteins after QCWZD treatment. Our results revealed that QCWZD can regulate JAK2/STAT3 signaling activation by decreasing the phosphorylation of colonic STAT3 and JAK2.

## 5. Conclusions

Our results suggest that QCWZD administration improves colitis by inhibiting M1 macrophage polarization *in vivo* and *in vitro*, and that this may be mediated by the JAK2/STAT3 signaling pathway. Our findings provide new evidence for the effect of QCWZD on intestinal inflammation regulation and the foundation for the development of novel macrophage-mediated therapeutic strategies. Nevertheless, future studies in patients with UC are warranted to fully elucidate the mechanisms underlying the effects of QCWZD on the gut.

## Figures and Tables

**Figure 1:** Major Qingchang Wenzhong decoction (QCWZD) components identified using high-performance liquid chromatography (HPLC). I: standard solution; II: QCWZD solution. (a) HPLC chromatogram of *Zingiber officinale* Roscoe, 1: 6-curcumin; (b) HPLC chromatogram of *Sanguisorba officinalis* L., 2: gallic acid; (c) HPLC chromatogram of *Coptis chinensis* Franch., 3a: epiberberine chloride; 3b: coptisine chloride; 3c: palmatine chloride; and 3d: berberine chloride; (d) HPLC chromatogram of *Panax notoginseng* (Burkill) F.H. Chen, 4a: notoginsenoside R1, 4b: ginsenoside Rg1, and 4c: ginsenoside Rb1; (e) HPLC chromatogram of *Strobilanthes cusia* (Nees) Kuntze, 5a: indigo and 5b: indirubin.

**Figure 2:** Qingchang Wenzhong decoction (QCWZD) treatment alleviates dextran sulfate sodium (DSS)-induced symptoms in mice. (a) Treatment procedure; (b) body weight; (c) disease activity index (DAI) score; (d) photograph of colon tissue; (e) colon length; (f) histological score; (g) hematoxylin and eosin (H&E) staining of colon tissue. ^#^*P* < 0.05, ^##^*P* < 0.01 versus the control group; ^∗^*P* < 0.05, ^∗∗^*P* < 0.01 versus the DSS group. *n* =4–6 for each group.

**Figure 3:** Qingchang Wenzhong decoction (QCWZD) treatment decreases the number of M1-like macrophages in the colon tissue of dextran sulfate sodium (DSS)-treated mice. (a) Protein expression levels of F4/80 and CD16/32 in the colon tissue of mice determined using immunofluorescence staining (F4/80, red; CD16/32, green; DAPI, blue); (b, e, f) mRNA levels of inducible nitric oxide synthase (iNOS), interleukin-6 (IL-6), and tumor necrosis factor-*α* (TNF-*α*) in colon tissue determined using real-time reverse transcription-quantitative polymerase chain reaction (RT-qPCR); (c, d) levels of TNF-*α* and IL-6 detected using ELISA. ^#^*P* < 0.05, ^##^*P* < 0.01 versus the control group; ^∗^*P* < 0.05, ^∗∗^*P* < 0.01 versus the DSS group. *n* =3–6 for each group.

**Figure 4:** Qingchang Wenzhong decoction (QCWZD) inhibits M1 polarization through the JAK2/STAT3 signaling pathway. (a–d) Protein levels of JAK2 and STAT3 in the colon tissue of mice determined using western blotting; *β*-actin was used as a reference. ^#^*P* < 0.05, ^##^*P* < 0.01 versus the control group; ^∗^*P* < 0.05 versus the DSS group. *n* =3 for each group.

**Figure 5:** Qingchang Wenzhong decoction (QCWZD) is non-toxic to macrophages. (a) RAW 264.7 cell viability test; (b, c) RAW 264.7 cell apoptosis test. ^#^*P* < 0.05 versus the control group. *n* =3 for each group.

**Figure 6:** Qingchang Wenzhong decoction (QCWZD) treatment inhibits the M1-like phenotype of RAW264.7 cells. (a) Inflammatory RAW264.7 cell (F4/80^+^CD16/32^+^) proportion using a Fluorescence Activated Cell Sorter; (b) M1 macrophage percentage; (c) inducible nitric oxide synthase (iNOS) expression levels detected using RTq-PCR; (d, e) concentration of interleukin-6 (IL-6), and tumor necrosis factor-*α* (TNF-*α*) in the supernatant tested using ELISA. ^##^*P* < 0.01 versus the control group; ^∗^*P* < 0.05, ^∗∗^*P* < 0.01 versus the LPS and IFN-*γ* group. *n* =3 for each group.

**Figure 7:** Qingchang Wenzhong decoction (QCWZD) inhibits the JAK2/STAT3 signaling pathway and M1 macrophage polarization. (a–d) RAW264.7 cells treated with 100 ng/mL lipopolysaccharide (LPS) and 10 ng/mL interferon-*γ* (IFN-*γ*) for 24 h, and 0.25 mg/mL and 0.125 mg/mL QCWZD, respectively, 2 h prior to treatment with LPS and IFN-*γ*. Protein levels of p-JAK2 and p-STAT3 in the colon tissue determined using western blotting; *β*-actin was used as a reference. ^#^*P* < 0.05, ^##^*P* < 0.01 versus the control group; ^∗^*P* < 0.05 versus the LPS and IFN-*γ* group. *n* =3 for each group.

**Table 1:** Primer sequence.

Genes	Forward (5′–3′)	Reverse (5′–3′)
iNOS	GGCAAACCCAAGGTCTACG	ACCTGCTCCTCGCTCAAGTT
TNF-*α*	CCCAGACCCTCACACTCAGATCATC	GTTGGTTGTCTTTGAGATCCATGCC
IL-6	GGAGTCACAGAAGGAGTGGCTAAG	AGTGAGGAATGTCCACAAACTGATA
GAPDH	CGTTGACATCCGTAAAGACCTC	ACAGAGTACTTGCGCTCAGGAG

**Table 2:** Content of the major indices in QCWZD.

Major indexes	Sample determination (mg/g)
6-curcumin	0.086
Gallic acid	0.868
Epiberberine chloride	1.638
Coptisine chloride	1.775
Palmatine chloride	3.032
Berberine chloride	13.235
Notoginsenoside R1	3.907
Ginsenoside Rg1	12.791
Ginsenoside Rb1	9.019
Indigo	7.045
Indirubin	0.52

## Data Availability

The datasets used and analyzed during the current study are available from the corresponding author upon reasonable request.
